The article "Flavonoids a Bioactive Compound from Medicinal Plants and Its Therapeutic Applications" was published in 2022. Journal: Biomed Res Int.

# Flavonoids a Bioactive Compound from Medicinal Plants and Its Therapeutic Applications

**DOI:** 10.1155/2022/5445291

**Published:** 2022-06-06

**Authors:** Arpita Roy, Ariba Khan, Irfan Ahmad, Saad Alghamdi, Bodour S. Rajab, Ahmad O. Babalghith, Mohammad Y. Alshahrani, Saiful Islam, Md. Rabiul Islam

**Affiliations:** ^1^Department of Biotechnology, School of Engineering & Technology, Sharda University, Greater Noida, India; ^2^Department of Life Sciences, School of Basic Sciences and Research, Sharda University, Greater Noida, India; ^3^Department of Clinical Laboratory Sciences, College of Applied Medical Sciences, King Khalid University, Abha, Saudi Arabia; ^4^Laboratory Medicine Department, Faculty of Applied Medical Sciences, Umm Al-Qura University, Makkah, Saudi Arabia; ^5^Medical Genetics Department, College of Medicine, Umm Al-Qura University, Makkah, Saudi Arabia; ^6^Civil Engineering Department, College of Engineering, King Khalid University, Abha 61413, Saudi Arabia; ^7^Department of Pharmacy, University of Asia Pacific, Dhaka, Bangladesh

## Abstract

Plants generally secrete secondary metabolites in response to stress. These secondary metabolites are very useful for humankind as they possess a wide range of therapeutic activities. Secondary metabolites produced by plants include alkaloids, flavonoids, terpenoids, and steroids. Flavonoids are one of the classes of secondary metabolites of plants found mainly in edible plant parts such as fruits, vegetables, stems, grains, and bark. They are synthesized by the phenylpropanoid pathway. Flavonoids possess antibacterial, antiviral, antioxidant, anti-inflammatory, antimutagenic, and anticarcinogenic properties. Due to their various therapeutic applications, various pharmaceutical companies have exploited different plants for the production of flavonoids. To overcome this situation, various biotechnological strategies have been incorporated to improve the production of different types of flavonoids. In this review, we have highlighted the various types of flavonoids, their biosynthesis, properties, and different strategies to enhance the production of flavonoids.

## 1. Introduction

Flavonoids are naturally occurring compounds that are present in the nascent parts of a plant. These are an abundant pigment along with chlorophylls and carotenoids that are present in almost all plants. They are known to provide fragrance and taste to fruits, flowers, and seeds. Flavonoids are low molecular weight polyphenolic phytochemicals secreted as a secondary metabolite in plants [1]. Secondary metabolites are produced in secondary pathways that synthesize compounds that are needed in trace amounts [2]. The secondary metabolites regulate primary pathways such as hormones, and coenzymes. During specific stress conditions, these act as toxins and antibiotics. In addition to their significant role in plants, they are important for human health because of various pharmacological activities. Some flavonoids are known as flower pigments that impart color aroma in flowers [3]. Flavonoids have been identified to have broad-spectrum effects in both microorganisms and animals with varied structures and functions. Since ancient times, the presence of flavonoids in plants has been identified, but their chemical structure was not known until the end of the nineteenth century [4]. In the early twentieth century, flavonoids and associated substances were chemically characterized in different plants and synthesized under laboratory conditions. Most of the interest was on their role as pigments, and the studies were mainly focused on the family of anthocyanins. Since then, more than 9,000 derivatives of flavonoids have been reported. A wide range of derivatives play an essential role in the integrity of plant structure, photoprotection from UV rays, reproduction, regulation of cell signaling, and physiology. Synthesis of flavonoids occurs from phenylalanine and malonyl coenzyme A. They are all structurally derived from parent compound flavones that are usually found in the cell sap of young tissues of plants.

The article "Flavonoids a Bioactive Compound from Medicinal Plants and Its Therapeutic Applications" was published in 2022. Journal: Biomed Res Int.

Flavonoids are biologically active phytochemicals that are ubiquitous in the plant kingdom which are being used in various herbal medicines for many years now. They constitute an essential part of our daily diet. They accumulate mainly in the edible parts of plants [5, 6]. Flavonoids are generally found in fruits, vegetables, grains, bark, stems, tea, and wine. There are multiple factors that are required to target the treatment of a complex chronic disorder, and in conventional treatment, this refers to polypharmacy. Therefore, it has to be emphasized that herbal medicines are a chemically complex blends containing multiple major and minor elements with multiple potent targets and processes. They are synthesized by the phenylpropanoid pathway and are derivatives of 2-phenylbenzyl-pyrone [7]. Flavonoids are a hydroxylated phenolic substance and are synthesized by plants in response to microbial infections. Many studies have been conducted on medicinal plants to explore their therapeutic potential to treat numerous diseases. Treatment with medicinal plants has been considered as safer due to their minimal to no side effects compared to conventional drugs. Medicinal plants show various potentials for the treatment of several diseases that are considered difficult to cure. Ayurveda has been using herbal drugs successfully for the prevention and suppression of various tumors for many years. Medicinal herbs have a positive impact as there are about half a million plants around the world and most of them have not yet been studied for medical purposes. Therefore, current and future studies on therapeutic activities can be effective in treating diseases

The article "Flavonoids a Bioactive Compound from Medicinal Plants and Its Therapeutic Applications" was published in 2022. Journal: Biomed Res Int.

## 2. Methodology

For this review paper, data has been collected by using different search engines which includes PubMed, ScienceDirect, Google Scholar, and ResearchGate.

## 3. Biosynthesis of Flavonoids

Biosynthesis of flavonoids starts with condensation of one molecule with three molecules of malonyl-CoA which yields chalcone by using chalcone synthase (CHS) (Figure 1). Then chalcone isomerization by using chalcone isomerase (CHI) leads to the formation of flavanone [8]. Then, it forms different classes of flavonoids.

## 4. Basic Structure and Type of Flavonoids

The basic structure of flavonoids (Figure 2) has a skeleton of diphenyl propane, which contains 15C atoms. Two 6-membered rings A and B linked with 3 carbon units which may or may be the part of the third ring. This 3-carbon ring is the heterocyclic oxygen-containing pyrene ring [9]. This basic structure of the flavonoid ring is also referred to as C6-C3-C6 structure [10]. Flavonoids are divided into various subgroups, which depend on the carbon of the C ring and the degree of oxidation of the B ring. Isoflavones are those in which the B ring is attached at position 3 of the C ring (Figure 3). Neoflavonoids have B rings attached to C rings at position 4 (Figure 4). And the others are where the B ring is attached to the C ring at position 2 and are further divided into different classes. And the other has opened the C ring [9].

### 4.1. Isoflavonoid

Isoflavonoids are a subgroup of flavonoids. They have a limited occurrence in plants and are mainly found in soya beans, in other leguminous plants, and in some microbes [11]. These compounds are able to prevent cancer and show an effect on cardiovascular and menopausal health [12]. They also have antioxidant effects on blood vessels. Isoflavonoids are also used as phytoestrogens because of the estrogenic activity shown by them in animal models [3].

### 4.2. Neoflavonoid

Neoflavonoids has a backbone of 4-phenylchromen with the absence of substituted hydroxyl group at the 2nd position. First, neoflavonoid, *Calophyllum inophyllum* was used in the year 1951. *Calophyllum inophyllum* was named and also found in the bark *of Mesua thwaitesii* [3].

### 4.3. Flavones

In flavones, the B ring is joined at 2 C to the C ring. The main flavonoids of this group are rutin, leutein, and luteolin glycosides. Other examples of flavonoids found in this group are apigenin and chrysin. The major dietary sources of flavones are fruits skin, red wine, buckwheat, red pepper, and tomato skin. They are found in several plants such as *Aloe vera*, *Bacopa moneirra* of the family Sarophulariaceae, *Mentha longifolica* of Lamiaceae family, and *Momordica charantia* of Cucurbitaceae [7].

The article "Flavonoids a Bioactive Compound from Medicinal Plants and Its Therapeutic Applications" was published in 2022. Journal: Biomed Res Int.

### 4.4. Flavonols

In flavonols, the B ring is attached to the C ring at 2 positions, and a hydroxyl group is attached to 3 positions of the C ring. The main examples of flavonols are quercetin, kaempferol, and galangin. Other ingredients are myricetin and tamarixetin. The main sources of flavonols are onion, red wine, olive oil, berries, and grapefruit [13]. They are found in plants such as *Acalypha indica*, *Azadirachta indica*, *Betula pendula*, and *Cannabis sativa* [14].

### 4.5. Flavanones

Flavanone is a significant class of flavonoids. Lemons, oranges, grapes, and citrus fruits are the main sources of flavanone (Felgines C, 2000). Naringin, naringenin, and hesperidin are some types of flavanones. Hesperidin is found in *Citrus medica* of the Rutaceae family [7].

### 4.6. Flavanonols

Flavanonols are the other classes of flavonoids. They have their basic structure in which the B ring is attached to the C ring at position 2 and the hydroxyl groups are attached at the 3rd position of the C ring and the 3rd and 4th positions of the B ring. An important compound of flavanonols is taxifolin [15].

### 4.7. Flavanols

Flavanols are also known as flavan-3-ols due to the presence of a OH group at position 3rd of C ring [16]. Like many flavonoids, there is an absence of double bonds between positions 2 and 3. Sources of flavanols are apples and tea. Catechin, epicatechin, epigallocatechin, glausan-3-epicatechin, and proanthocyanidins are included under flavanols [17]. Plant source of flavanols includes *Brysonima crassa* [18].

### 4.8. Chalcones

Chalcones include phloretin and chalconaringenin [3]. They are characterized by the absence of C ring, or we can say there the C ring has an open structure. Therefore, they are also known as open-chain flavonoids. Different structure of different flavonoids are given in Figure 5.

## 5. Function of Flavonoids in Plants

Flavonoids play a wide number of important roles in plants (Figure 6). Flavonoids acts as signaling molecules, detoxifying agents, phytoalexins and hepls in the stimulation of seed germination, temperature acclimatization, and provide drought resistance. Flavonoids also reduce reactive oxygen species in plant tissue, which are generally generated due to infection or UV irradiation. Another important role they play is in the fragrance, color, and taste of fruits, flowers, or seeds. This fragrance and color attract pollinators that help pollination and dispersal of seeds [20].

The article "Flavonoids a Bioactive Compound from Medicinal Plants and Its Therapeutic Applications" was published in 2022. Journal: Biomed Res Int.

### 5.1. Protect against Radiation

Flavonoids have the property of UV absorption, which is why they are considered to play a role in the protection of plants from UV radiation. Some of them act as free radical scavengers such as reactive oxygen species (ROS) and chelating metals [21]. UV light induces the formation of flavonol due to the presence of OH in the third position of the flavonoid backbone, and this is the main reason that is responsible for its chelating property of metal ions like iron, zinc, aluminum, and copper, and this property of them inhibits the formation of free radicals and reduces ROS that have already been produced; this was evident in some plants like *Petunia*, *Arabidopsis*, grapevine, and wild privet.

### 5.2. Protect against Infection

Flavonoids give protection to plants from pathogens and herbivores. They secrete substances such as phytoalexins and lignins that act as a barrier to prevent the spread of pathogens and regulate the expression of these genes that produce protective metabolites like flavonols. Legumes such as soya bean and chickpea produce isoflavonoids which play an important role in defense against pathogens. Vesitol, which comes from the class of isoflavans, is the main phytoalexin synthesized by lotus species. The C-glycosyl flavones maysin and other compounds such as apimaysin and methoxymaysin are secreted by maize in response to its pest corn earworm and interfere with its amino acid metabolism in the guts and are converted into very toxic quinones. These quinones bind to the -SH and -NH2 of proteins and amino acids and hence reduce their availability [21].

### 5.3. Fertility and Reproduction

Flavonoids give color and fragrance to flowers and fruits in different plant species and attract pollinators. These pollinators help to remove and grow seeds and plants. The most important and major class of flavonoids that play a role in plant pollination is the anthocyanins present in flowers and fruits. Production of seed fruits and low level of anthocyanidin in tobacco is also achieved by blocking the pathway of rutin, a type of flavonol. Parthenocarpy is achieved by chalcone synthase gene silencing and by applying the flavonol quercetin and kaempferol these processes can be reversed. Thus, in this way, flavonoids play an essential role in the fertility and reproduction of plants [21].

### 5.4. Rhizosphere

Flavonoids also play an important role in the rhizosphere region of the roots of the plant by stimulating spore germination and chemoattraction of rhizobia, and they also amplify the expression of nod genes. Plant secretes flavonoids in response to infection by rhizobia such as *Azorhizobium*, *Bradyrhizobium*, *Mezorhizobium*, and *Sinorhizobium* as a result of which the plant oozes out flavonoids [22]. When these bacteria interact with the plants, they form a nodule and the bacteria remain inside the nodule as a bacteroid, this process results in the N2 fixation [22].

The article "Flavonoids a Bioactive Compound from Medicinal Plants and Its Therapeutic Applications" was published in 2022. Journal: Biomed Res Int.

### 5.5. Extraction Processes for Flavonoids

#### 5.5.1. Conventional Technique

There are various methods used for the extraction of flavonoids. These include percolation, maceration, hydrodistillation, Soxhlet reflux, and soaking. Among these methods, Soxhlet is the simplest, easiest to use, and most widely used method used for the extraction of flavonoids. Water infusion and marceration are the old extraction processes to adopt ethanol, acetone, and methanol usage for the extraction of flavonoids which they are still being used. Various factors are taken into account when using conventional methods. These factors are time, solvent type, mass to volume ratio, temperature, and particle size. Of the various solvents used in these extraction processes, ethanol and methanol are the most commonly used.

#### 5.5.2. Enzyme-Assisted Technique

The enzyme-assisted method is an alternative method to the conventional method. This uses the specificity of enzymes and their regioselectivity. In this method, less solvent is used compared to conventional methods [23]. Enzymes from various sources like fungi, bacteria, plants, fruits, and vegetables breakdown the cell wall, and this can increase the cell wall permeability and thus increases the extraction yield. Cello-bio-hydrolases, *β*-glucosidases, and endo- and exo-glucanases hydrolyze cellulase and increase cell permeability. Hemicellulose chains are degraded by the use of the enzymes pectin lyase, pectate lyase, and endo- and exo-polygalactouronases. Factors like treatment time, pH, and temperature and the amount of the enzyme are considered while using this method [23].

#### 5.5.3. Extraction Using Ultrasound-Assisted Technique

100 g of lotus leaves suspended in ethanol of concentration 40-80% and soaked in it for about 4 h in ultrasonic light for 15-40 min in ultrasound cleaner. From this, a deep brown extract was obtained, which was then filtered using the filter. This filter is then absorbed by D101 macroporous absorptive resin column at a speed of about 20 ml/min. This column is then eluted with dH2O to make this liquid colorless and then eluted with 80% ethanol. Then using a rotatory evaporator, cooled elutant was evaporated and pressure was reduced in order to obtain the flavonoids. In this extraction method, it was found that the extraction yield of flavonoids increased when ethanol was used in conc. 40-70%, but beyond 70%, the yield reduces [24].

The article "Flavonoids a Bioactive Compound from Medicinal Plants and Its Therapeutic Applications" was published in 2022. Journal: Biomed Res Int.

#### 5.5.4. Supercritical Fluid Extraction Method

Fluids that are above their thermodynamically critical temperature and pressure are known as supercritical fluids. Under these conditions, the viscosity decreases, and the diffusivity of the solvent increases. CO2, because of its flammable, nontoxic, cheap, and easy-to-use properties, is the most widely used solvent that is used in extraction methods. Low temperature which maintains the integrity of the products, high volatility of the solvent that reduces waste, and the separation of volatile from nonvolatile compounds are the advantages of using the supercritical fluid extraction method [23].

## 6. Therapeutic Properties of Flavonoids

Flavonoids have anti-inflammatory, antimutagenic, antiallergic, antiviral, and anticarcinogenic properties [23] (Figure 6). They also process therapeutic and cytotoxic activity. Flavonoids are inhibitors of various enzymes such as xanthine oxidase (XO), cyclooxygenase (COX), lipoxygenase, and phosphoinositol-3-kinase [25]. Flavonoids give color and aroma to the flowers; in fruits, they attract pollinators; and as a consequence, the pollinators help in seed dispersal and spore germination and seed growth. They protect the plant from biotic and abiotic stress and function as signal molecules, detoxing agents, UV filters, allopathic compounds, and phytoalexins and play an important role in drought resistance and tolerance to freezing [3].

### 6.1. Antioxidant Activity

Antioxidants are compounds which protect plants, animals, and humans against the effect of reacting oxygen species (ROS). Flavonoids act as an antioxidant by suppressing ROS formation either by inhibition of the enzyme or by chelating the trace elements involved in free radical generation, by scavenging ROS, or by upregulation or protection of antioxidant defenses [26]. The appearance, position, structure, and number of attached sugar units play an important role in antioxidant activity. The antioxidant activity of flavonoids is the most important activity.

### 6.2. Antiviral Activity

Flavonoids such as flavon-3-ol, flavones, and flavanones are effective against viral infection compared to flavones. Flavon-3-ol is more effective against HIV 1 and HIV 2 immunodeficiency [7]. According to studies, other flavonoids which show antiviral activity include quercetin, hespertin, and naringin. They possess antidengue activity [27]. These antiviral flavonoids help in the inhibition of various enzymes involved in the virus life cycle. Various studies have also focused on apigenin, vitexin, and their derivatives which were found to be active against many viruses such as hepatitis C virus, herpes simplex virus 1 (HSV-1), human hepatitis A and B and C virus, rhesus rotavirus (RRV), and influenza viruses [28].

The article "Flavonoids a Bioactive Compound from Medicinal Plants and Its Therapeutic Applications" was published in 2022. Journal: Biomed Res Int.

### 6.3. Antimicrobial Activity

Various studies have shown that flavonoids are secreted by plants in response to bacterial infection. Flavonoids such as apigenin, galangin, flavone glycosidase, and chalone have been proved to show antibacterial properties by Cushnie and Lamb [29]. A wide variety of nonflowering medicinal plants and flowering plants show antibacterial activity by a large number flavonoid. *Asplenium nidus nidus* L. contains gliricidin 7-O-hexoside, and quercetin-7-O-rutinoside is a fern that gives protection for three pathogens, namely, *Proteus mirabilis* Hauser, *Pseudomonas aeruginosa* (Schroeter), and *Proteus vulgaris* [30]. Plants that are involved in traditional and dietary medicine also secrete various flavonoids and phenolic compounds. Nutmeg (*Myristica fragrans* Houtt.) is a flavoring agent used in India and other countries in Southeast Asia. Nutmeg activities can help to recuse a large number of species related to oxidative stress [14]. Flavonoids are also used in skin acne problems and show antibacterial activity for *P. acnes*. Chlorine-containing chloroflavin is the first flavonoid antibiotic against fungi. The peeling of oranges also contains several flavonoids that have fungistic activity against *Deuterophoma tracheiphila*. Myricetin, a flavonoid, inhibits the growth of multidrug resistance bacteria *Burkolderia cepcia* and inhibits protein synthesis by *B. cepcia* [31].

### 6.4. Cardioprotection

Many studies have shown the effectiveness of flavonoids in cardioprotection. Hypertension and atherosclerosis can be prevented by the usage of flavonoids. These flavonoids reduce atrial pressure, enhance the vasorelaxant process, and prevent endothelial dysfunction. Endothelial dysfunction is a leading cause of cardiovascular disease and is the major complication of atherosclerosis and arterial thrombus formation. Endothelium-dependent vasorelaxation is exerted by *anthocyanin delphinidin*. Atherosclerosis development starts with the oxidative modification of low-density lipoproteins by free radicals. Scavenger receptors take this modified LDL and lead to the formation of cells [32]. Cardioprotection is achieved by the activity of quercetin and quercetin glycosides by protecting the LDL from oxidative modification. The antioxidant activities of polyphenolics may have significant benefits for health. This is due to the ability of polyphenols to transfer electron chelation of ferrous ions, and they also scavenge reactive oxygen species (ROS), and due to this, they are used in the protection of chronic cardioactivity [33].

The article "Flavonoids a Bioactive Compound from Medicinal Plants and Its Therapeutic Applications" was published in 2022. Journal: Biomed Res Int.

### 6.5. Antidiabetic Activity

Flavonoids also possess antidiabetic activity by regulating carbohydrate digestion, insulin secretion, insulin signaling, glucose uptake, and adipose deposition [34]. They target multiple molecules that are involved in the regulation of several pathways such as improvement of *β*-cell proliferation, promoting insulin secretion, apoptosis reduction, and improving hyperglycemia by regulating glucose metabolism in the liver [35]. In US, a study was conducted where 200,000 women and men were suppelemented with dietary flavonoids. The study confirmed that a higher consumption of anthocyanins from blueberries, apples and pears, reduce the risk of diabetes. It was hypothesized that the majority of flavonoids bioactivity occurs due to their hydroxyl group, *α*, and *β* ketones [36].

### 6.6. Anticancer Activity

Studies have been reported that flavonoids are able to inhibit tumor cell proliferation by inhibiting formation of ROS and repression of xanthine oxidase, cyclooxygenase-2, and 5-lipoxygenase enzymes, which play important role in tumor promotion and development [37]. Flavonoids possess wide range of anticancer effects. In a study, it was reported that isorhamnetin and acacetin can inhibit human breast cancer proliferation [38]. In another study, kaempferol showed antiproliferative and apoptosis activity against breast (MCF-7) cancer, human osteosarcoma, stomach (SGC-7901), and lung (A549) carcinoma cells [39]. Another study reported that hesperidin can reduce progression of cell cycle in osteosarcoma MG-63 cells and induce apoptosis in various cancer cells like ovary, breast, prostate, and colon cancer cells [40]. Additionally, hesperidin shows antitumor and hepatoprotective effects against the development of hepatocellular carcinoma [40]. Cyanidin also showed inhibition of proliferation and induction of apoptosis in human epithelial colorectal adenocarcinoma cells [41].

## 7. Strategies to Enhance Flavonoid Production

Production of flavonoids can be improved via numerous techniques (Figure 7). One of the most effective tools is elicitation and feeding of precursors. In a study, the elicitation of hairy root culture by chitosan from seven species of *Psoralea* was found to enhance the production of flavonoids such as daidzein and coumestrol [42]. When the result of flavonoid production from hairy root culture and callus culture was compared, it was found that flavonoid production from hairy root culture was higher [42]. In another study, methyl jasmonate was used to improve flavonoid production in a cell suspension culture of *H. perforatum*. It was found that 100 *μ*mol/L of methyl jasmonate treatment resulted in maximum production of flavonoid, i.e., 280 mg/L, which was 2.7 times higher than the control culture [43]. Quercetin and rutin production from hairy root culture of *F. tataricum* has been enhanced to 47.13 mg/l, which was about 3.2 times higher than that of control culture, i.e., 14.88 mg/L [44]. Shaw et al. [45] elicited an in vitro culture of *Hordeum vulgare* using CuONP and found that the leaves showed a significant enhancement of flavonol levels (~1.2 times more than the control) after 20 days of treatment. Fazal et al. [46] reported the treatment of silver and gold nanoparticles in callus cultures of *Prunella vulgaris*. They found that silver gold nanoparticles in the ration of 1 : 3 in combination with NAA enhanced flavonoid accumulation, i.e., 6.71 mg/g Dw. Genady et al. [47] used the treatment with copper sulfate nanoparticles in *O. basilicum* and found an enhanced flavonoid content. In a study, hairy root of *Dracocephalum kotschyi* was treated with iron oxide nanoparticles which showed enhanced flavonoid accumulation [48]. The cell suspension culture of *Momordica charantia* was treated with silver nanoparticles synthesized by *Bacillus licheniformis* [49], and it was found that the elicitation increased the concentration of flavonoids present in the plant, such as quercetin, kaempeferol, myricetin, catechin, naringenin, rutin, and biochanin A. A study showed that *Cucumis anguria* hairy root culture treatment with silver nanoparticles enhanced the production of flavonoids [50]. Singh et al. [51] reported the highest flavonoid production, i.e., 23.076 ± 5.128 mg QE/g extract after 20 days of CuONP treatment in case of *Withania somnifera*. Chung et al. [52] reported the treatment of *Gymnema sylvestre* cell suspension culture with copper oxide nanoparticles and found that it increased the production of total flavonoid content by two times. Nourozi et al. [53] reported the treatment of iron oxide nanoparticles in hairy root culture of *Dracocephalum kotschyi* that improved flavonoid production. Herbal products and natural phytochemicals, like flavonoids, flavonols, and other bioactive compounds, exhibit health-promoting effects. Evidence suggests that these metabolites have the potential to protect different cells from oxidative damage [54, 55]. A study reported that foliar application of jasmonic acid at a concentration of 0.25 mM resulted in improved antioxidant responses including flavonoid and anthocyanin production in *Jatropha curcas* [56]. Another study reported accumulation of flavonoids in *Isatis tinctoria* L. hairy root culture which was elicited by 179.54 *μ*M methyl jasmonate, and it increased 11.21-folds as compared with controls [57].

The article "Flavonoids a Bioactive Compound from Medicinal Plants and Its Therapeutic Applications" was published in 2022. Journal: Biomed Res Int.

## 8. Toxicological Evaluation of Flavonoids

Toxicological evaluation of flavonoids is also an important aspect which needs to be taken into consideration. A study reported the evaluation of safety and toxicity of chrysin (plant flavonoid) after acute and subchronic oral administration in rats. It was found that acute oral administration of chrysin (5000 mg/kg) showed 40% mortality. In the subchronic toxicity study, daily oral administration of chrysin (1000 mg/kg) showed suggestively decreased body weight, whereas liver weight was improved significantly in male rats. Significant increase in renal and hepatic oxido-nitrosative stress was also observed, and no significant change in electrocardiographic, hemodynamic, the left ventricular function, and lung function test was found [58]. In a study, subchronic toxicity and genotoxicity of a flavonoid-rich extract from Maydis stigma was evaluated in mice. It was found that all animals survived until the planned necropsy, and no statistically significant or toxicologically relevant differences were observed in any of the treatment groups as compared to control one [59]. A study was conducted to investigate preclinical safety of four flavonoids, i.e., naringin, naringenin, hesperidin, and quercetin. Cytotoxicity was evaluated against VERO and MDCK cell lines, and it was found that quercetin was slightly more cytotoxic on cell lines than the other citroflavonoids. All flavonoids showed an LD50 value more than 2000 mg/kg, which categorizes them as low-risk substances. Similarly, predicted LD50 was LD50 more than 300 to 2000 mg/kg for all flavonoids as acute toxicity assay estimated and suggests that all these flavonoids did not show significant toxicological effects, and they were classified as low-risk, useful substances for drug development [60].

## 9. Conclusions and Future Prospects

Flavonoids are secondary metabolites which are secreted by plants. They provide various therapeutic applications for mankind which include cardioprotection, antidiabetic, and antiviral activity, as well as protection for plants in response to stress. They also play an important role in plant reproduction and fertility and in atmospheric nitrogen fixation. In summary, the valuable role of flavonoids for human health has generated increased consumption of these compounds. Vegetables, flowers, and seeds are rich source of flavonoids. The recognition of natural flavonoids as a good, safer source of antioxidants opens new perspectives to explore more of these compounds, focusing on new structures using new methodologies and technologies and exploiting other new natural sources. This review provides an overview of the role of flavonoids in plants, extraction procedures, and their therapeutic application for the benefit of humanity. Further production of different flavonoids using in vitro culture systems has been discussed.

The article "Flavonoids a Bioactive Compound from Medicinal Plants and Its Therapeutic Applications" was published in 2022. Journal: Biomed Res Int.

## Figures and Tables

**Figure 1:** Flavonoid synthesis.

**Figure 2:** Basic structure of flavonoids.

**Figure 3:** Structure of isoflavones.

**Figure 4:** Structure of neoflavonoids.

**Figure 5:** Structures of flavonoids [19].

**Figure 6:** Function of flavonoids in plants.

**Figure 7:** Strategies to enhance flavonoid production.

## Data Availability

All data used to support the findings of this study are included within the article.
